# Metagenomic Sequencing Analysis for Acne Using Machine Learning Methods Adapted to Single or Multiple Data

**DOI:** 10.1155/2021/8008731

**Published:** 2021-11-13

**Authors:** Yu Wang, Mengru Sun, Yifan Duan

**Affiliations:** Beijing Key Laboratory of Big Data Technology for Food Safety, School of Artificial Intelligence, Beijing Technology and Business University, Beijing 100048, China

## Abstract

The human health status can be assessed by the means of research and analysis of the human microbiome. Acne is a common skin disease whose morbidity increases year by year. The lipids which influence acne to a large extent are studied by metagenomic methods in recent years. In this paper, machine learning methods are used to analyze metagenomic sequencing data of acne, i.e., all kinds of lipids in the face skin. Firstly, lipids data of the diseased skin (DS) samples and the healthy skin (HS) samples of acne patients and the normal control (NC) samples of healthy person are, respectively, analyzed by using principal component analysis (PCA) and kernel principal component analysis (KPCA). Then, the lipids which have main influence on each kind of sample are obtained. In addition, a multiset canonical correlation analysis (MCCA) is utilized to get lipids which can differentiate the face skins of the above three samples. The experimental results show the machine learning methods can effectively analyze metagenomic sequencing data of acne. According to the results, lipids which only influence one of the three samples or the lipids which simultaneously have different degree of influence on these three samples can be used as indicators to judge skin statuses.

## 1. Introduction

Microbes are invisible to our naked eyes but are major residents living on the earth. Any environment which can be imagined, such as air dust, surface soil, underground rocks, waters systems, and other natural environments, as well as animals including humans, may have some certain microbes. The ecological community of microbes which lives at a certain part of the host body is referred to as a microbiota. The microbiota usually includes bacteria, archaea, microscopic eukaryotes, and viruses [1, 2]. The collection of genomes and genes which exist in the microbes is called the microbiome [3, 4]. They have significant influence on the environment or their host via complex interactions [5–7].

In a sense, the human body is not an individual organism but a complex community or symbiotic organism of human cells and various microbial species. Earlier research on human microbes focused on specific pathogens which caused human diseases. As the study is deepened step by step, especially in the past decade, researchers have found that (1) microbes inside and outside the human body maybe not only are pathogenicity, but also are a beneficial probiotic to the host. (2) In most cases, microbes living together with the host play an important role as a whole [4]. Studies have shown that human health can be assessed by research and analysis of the human microbiome [8, 9].

The traditional methods of studying the microbiome are based on independent cultivation of each microbial strain. Then, its characteristics and functions are studied. The related research results give us a lot of knowledge and inspiration about microbes. Limitations, however, also usually exist. On the one hand, it has been reported that 99% of microbes cannot be isolated and cultured [10, 11], which means that a large number of microbes cannot be studied using separation methods. On the other hand, microbes of microbiota tend to live and function as members of a system rather than a group of isolated microbes [12]. As a result, researchers began to look for new ways to obtain indirectly genomic information from microbial communities. Therefore, metagenomics came into being. Metagenomics refers to the sum of genome information for all species in an environmental microbiota. With the development of next-generation sequencing (NGS) technology, it is now very convenient to use metagenomic sequencing to study microbes. Due to the importance of microbes to human health, more and more researchers have begun to use metagenomic sequencing to study human microbes [13, 14]. With the rapid development of high-throughput sequencing technologies and the substantial reduction of sequencing costs, metagenomic sequencing has become a promising pathogen detection method for accurate diagnosis of infectious diseases [15]. Fan et al. [16] performed metagenomic sequencing for the cerebrospinal fluid of 4 patients with suspected central nervous system infection, and Brucella was detected within 48 hours. However, if the above results were verified by polymerase chain reaction and Sanger sequencing, the patient's cerebrospinal fluid needed be cultured for 7 days, which indicated that metagenomic sequencing was more rapid, efficient, and accurate in detecting pathogens than the culture method. Metagenomic sequencing, as a fast, low-cost, and high-throughput pathogen DNA sequencing technology, has high efficiency and accuracy for detection and has been used to detect various pathogen infections, which demonstrates that metagenomic sequencing can effectively guide clinical treatment [17]. At present, classification and prediction methods based on machine learning have been successfully applied to many fields such as complex text sentiment analysis, satire identification, and other difficult predictions and classifications [18–20]. In recent years, so much work on machine learning applied to metagenomics has done. Machine learning can be applied to the clustering, binning of the metagenomic data, comparative metagenomics and gene prediction, and so on [21–23]. Principal component analysis is used to obtain the bacteria which have main effect on the gingivitis by analyzing the data of gingivitis and healthy gums [24]. In the human gut metagenomics study of type 2 diabetes, the gene cluster which is found by correlation analysis represents the difference of the samples [25].

The skin is the most exposed organ in the body, and it is also the front line that protects various tissues and organs in the body from physical and chemical damage or damage of pathogenic microorganisms. Globally, the prevalence of skin diseases is increasing. According to statistics, acne is the most common skin disease in the world. Acne is a benignly evolutionary and chronic skin disease characterized by the inflammatory process of the hair follicles and attached sebaceous glands [26–29].

Acne mainly occurs in the facial and thoracodorsal areas and other seborrheic areas [30]. And its manifestations are polymorphic, ranging from blackheads, pimples, pustules to more severe statuses such as nodules, cysts, and pustules [29, 31]. The long course of acne and high recurrence rate badly affect the patient's appearance. Simultaneously acne can reduce the sense of beauty and even can cause mental illnesses such as low self-esteem, negative emotion, anxiety, and depression [32–34]. Therefore, the study and treatment of acne is an important and widely studied issue in the dermatology field. Acne's pathogenesis is complex. At present, many researchers have studied the role of bacteria in the pathogenesis of acne, such as Propionibacterium acnes (P. acnes), Staphylococcus epidermidis (S. epidermidis), and Staphylococcus aureus (S. aureus) [23, 35–38]. However, whether these bacteria are the main pathogens of acne is also controversial at present [38–41].

Due to the effective application of machine learning to metagenomic data, we attempt to analyze the metagenomic sequencing data of acne using machine learning methods. In this article, we obtained metagenomic sequencing data from the three skin statuses including face skin of healthy people, healthy face skin, and diseased face skin of acne patients. Principal component analysis (PCA) and kernel principal component analysis (KPCA) methods are used to find the corresponding lipids which largely contribute to the status of each kind of skin. In addition, multisets of canonical correlation analysis (MCCA) method are used to obtain lipids which can effectively differentiate the above three different skin statuses.  Figure 1 is the framework diagram of the proposed method.

The rest of this paper is organized a follows. Firstly, the Material and Methods are detailedly described in Section 2. Then, extensive experiments of metagenomic sequencing data of acne are presented in Section 3. Finally, a conclusion is drawn in Section 4.

## 2. Materials and Methods

### 2.1. Sample Collection

The data collection process for this experiment was as follows. For 35 acne patients, both infected cells and healthy cells of the face skin are collected. For 35 normal control (NC) who do not suffer from the acne, their healthy skin cells from the face are collected. The chromatographic apparatus applied was a set of Waters ACQUITY UPLC I-Class (Waters Corporation, Milford, Massachusetts, USA). The flow rate was maintained at 0.3 mL/min. The injection volume was 2.0 *μ*L. During UPLC runs, the injector needle was washed with the mobile phase. The eluent outlet was connected to QTOF-MS for entity detection and characterization. High-resolution mass measurements were performed with a Waters Xevo G2-XS QTOF-MS (Waters Corporation, Milford, Massachusetts, USA) equipped with an electrospray ionization (ESI) interface operating in the positive ion mode. Entities eluted from the UPLC system were introduced into the QTOF-MS apparatus at the operating chromatographic flow rate. Nitrogen was used as the nebulizing and desolvation gas. UPLC-QTOF-MS data were collected as raw data by Masslynx 4.1 (Waters Corporation, Milford, Massachusetts, USA). Therefore, three sample sets for this experiment including the patient's diseased skin (DS) samples, the patient's healthy skin (HS) samples, and NC samples are obtained. Each sample set has 35 volunteers, and each volunteer was extracted 2520 sequence data.

### 2.2. Principal Component Analysis

Principal component analysis (PCA) is a common means in data analysis. It is hoped that fewer variables can be used to interpret most of variables in the original data, and the main feature components of the data are extracted.

Suppose the sample set *X* includes *m* samples, and each sample is *n*-dimensional vector. At the same time, the sum of these *m* samples is 0 as shown in Equations (1) and (2).

(1) $$\begin{array}{c} X_{n\times m}=\left(x_{1},x_{2},\cdots ,x_{m}\right), \end{array}$$

(2) $$\begin{array}{c} \overset{m}{\underset{i=0}{\sum }}x_{i}=0. \end{array}$$

Suppose the new coordinate system is *W*_*n*×*n*_ = (*w*_1_, *w*_2_, ⋯, *w*_*n*_) after the transformation of projection, where *w*_*i*_ is an orthonormal basis. The original data sample is projected to a new coordinate system. The projection rule is shown in Equation (3).

(3) $$\begin{array}{c} Z_{n\times m}=W_{n\times n}^{T}\times X_{n\times m}. \end{array}$$

For separating all samples as far as possible after projection, the variance of these samples after projection should be maximized. Therefore, the optimized objective function is shown in Equations (4), where *I* is the unit vector.

(4) $$\begin{array}{c} \underset{W}{\max tr}\left(W^{T}{XX}^{T}W\right)s.t.W^{T}W=I. \end{array}$$

The Lagrange multiplier method is used to solve the equation, and the objective function is shown as follows.

(5) $$\begin{array}{c} J\left(W\right)=tr\left(W^{T}{XX}^{T}W+\lambda \left(W^{T}W-I\right)\right). \end{array}$$

The derivative of the above equation is obtained and shown in Equation (6).

(6) $$\begin{array}{c} {XX}^{T}W=\lambda W. \end{array}$$

It can be seen from the above equation that for finding the eigenspace *W*_*n*×*n*_, the corresponding eigenvalues and eigenvectors of the covariance matrix should be calculated. However, the eigenspace obtained is still *n*-dimensional and has not achieved the goal of dimensionality reduction. Therefore, the eigenvalue *λ* is arranged in descending order, and a reconstruction threshold *t*_1_ is selected using the following equation.

(7) $$\begin{array}{c} \frac{\sum_{i=1}^{k}\lambda_{i}}{\sum_{i=1}^{n}\lambda_{i}}\geq t_{1}. \end{array}$$

Then, the eigenspace *W*_*n*×*k*_ = (*w*_1_, *w*_2_, ⋯, *w*_*k*_)(*k* < *n*) composed of *k* eigenvectors can be determined. The information contained in the discarded part is often related to noise. Therefore, discarding this part of information can improve the experimental effect to a certain extent. In general, when the reconstruction threshold *t*_1_ reaches 85%, it is considered that the found principal components have large effect on the sample set.

### 2.3. Kernel Principal Component Analysis

Compared with PCA, kernel principal component analysis (KPCA) can mine the nonlinear information contained in the data set. In KPCA, a kernel function is introduced and used to calculate the kernel matrix *K* of the input data. Gaussian kernel is selected as the kernel function, so the kernel matrix *K* is described as

(8) $$\begin{array}{c} K_{i\times j}=e^{{\left\|X_{i}-X_{j}\right\|}^{2}/2\sigma^{2}}. \end{array}$$

Then, eigenvalues and eigenvectors of the kernel matrix *K* are calculated. After arranging the eigenvalues from the largest to the smallest, the reconstruction threshold *t*_1_ should be set to determine the eigenspace *W*. In our experiment, the reconstruction threshold *t*_1_ is set 95% and 99% for both PCA and KPCA.

### 2.4. Multiset Canonical Correlation Analysis

Since the PCA and KPCA methods only can analyze a kind of sample set. In order to obtain lipids which better distinguish three samples, a multiset canonical correlation analysis (MCCA) method is used. MCCA is used to analyze the relationship between multiple sets of data. The main idea of MCCA is that when the correlation coefficient *β* between several sample sets is maximum, the typical variable *w*_*i*_ corresponding to each sample set is found. Given the number of sample sets is *u*, and each sample set includes *N* samples, the objective function is described as

(9) $$\begin{array}{c} \arg\max\beta =\overset{u}{\underset{\begin{array}{c} k,l=1\\ k\neq l \end{array}}{\sum }}w_{k}^{T}\underset{ij}{\sum }w_{l}\left(k\neq l\right)s.t.\overset{u}{\underset{k=1}{\sum }}w_{k}^{T}\underset{ij}{\sum }w_{l}=1, \end{array}$$

where ∑_*ij*_ = *x*_*k*_^*T*^ · *x*_*l*_.

Using the Lagrange multiplier method for the objective function, the following equation can be obtained:

(10) $$\begin{array}{c} \left(C-D\right)w=\beta Dw, \end{array}$$

where $C=\left(\begin{array}{ccc} x_{1}x_{1}^{T} & \cdots & x_{1}x_{N}^{T}\\ \vdots & \ddots & \vdots \\ x_{N}x_{1}^{T} & \cdots & x_{N}x_{N}^{T} \end{array}\right)$ and $D=\left(\begin{array}{ccc} x_{1}x_{1}^{T} & \cdots & 0\\ \vdots & \ddots & \vdots \\ 0 & \cdots & x_{N}x_{N}^{T} \end{array}\right)$.

Then, the influential lipids can be found by the means of the typical variable *w*_*i*_.

### 2.5. Feature Selection

Data can be reconstructed using PCA and KPCA as shown in Equation (11).

(11) $$\begin{array}{c} Y_{k\times m}=W_{n\times k}^{T}\times X_{n\times m}. \end{array}$$

The new data after dimension reduction is *Y*_*k*×*m*_ = (*y*_1_, *y*_2_, ⋯, *y*_*m*_). In this way, *n*-dimensional data in the original data *X* is reduced to the *k*-dimensional data. The obtained *Y* is already the data in another spatial dimension and not the lipid information of the original data. Therefore, based on the relevant knowledge of mathematical statistics, a method is proposed to map the eigenspace to the input space in this paper.

First of all, the position information of several basis space components *w*_*j*×*p*_ which have the greatest influence on the new data *Y* is counted, corresponding to the lipids of the original data. Then, the frequency of each original data in the same eigenvector is calculated, and weights are added according to its eigenvalues. Finally, the frequencies and weights of the original data counted by all eigenvectors are multiplied, and the product is summed if it is the same original data. All of products are arranged in descending order, and the maximum *k* results are lipids that have greater impact on acne.

In Equation (11), each element in *Y* is calculated as shown in Equation (12):

(12) $$\begin{array}{c} \left[\begin{array}{cccc} y_{1\times 1} & y_{1\times 2} & \cdots & y_{1\times m}\\ y_{2\times 1} & y_{2\times 2} & \cdots & y_{2\times m}\\ \cdot & \cdot & \cdots & \cdot \\ \cdot & \cdot & \cdots & \cdot \\ \cdot & \cdot & \cdots & \cdot \\ y_{k\times 1} & y_{k\times 2} & \cdots & y_{k\times m} \end{array}\right]=\overset{n}{\underset{j=1}{\sum }}\left[\begin{array}{cccc} w_{j\times 1}\cdot x_{j\times 1} & w_{j\times 1}\cdot x_{j\times 2} & \cdots & w_{j\times 1}\cdot x_{j\times m}\\ w_{j\times 2}\cdot x_{j\times 1} & w_{j\times 2}\cdot x_{j\times 2} & \cdots & w_{j\times 2}\cdot x_{j\times m}\\ \cdot & \cdot & \cdots & \cdot \\ \cdot & \cdot & \cdots & \cdot \\ \cdot & \cdot & \cdots & \cdot \\ w_{j\times k}\cdot x_{j\times 1} & w_{j\times k}\cdot x_{j\times 2} & \cdots & w_{j\times k}\cdot x_{j\times m} \end{array}\right]. \end{array}$$

Each element *y*_*p*/*q*_ is the sum of *n* multipliers, and each multiplier is the product of the basis space component and the original data. For each element *y*_*p*×*q*_, *n* multipliers are arranged in descending order during the process of accumulation, and each multiplier is expressed as *w*_*j*×*p*_^count^ · *x*_*j*×*p*_, count ∈ [1, *n*]. The larger the number count is, the smaller the value is. The threshold value *t*_2_ is selected to satisfy Equation (13), and the position information of these l base space components *w*_*j*×*p*_ which maximize the multiplier is recorded.

(13) $$\begin{array}{c} \frac{\sum_{\text{count}=1}^{l}w_{j\times p}^{\text{count}}\cdot x_{j\times q}}{\sum_{\text{count}=1}^{n}w_{j\times p}^{\text{count}}\cdot x_{j\times q}}\geq t_{2}. \end{array}$$

Because each eigenvalue corresponding to eigenvector is different, the position information of basis space components obtained in each eigenvector must be divided into a group. The position information of basis space component corresponds to the original data, and then, the frequencies *f*_*i*×*j*_(*i* ∈ [1, *k*]) of different original data in each group are, respectively, calculated, where *j* represents the space component location information. Equation (14) is used to calculate the projects after adding weight.

(14) $$\begin{array}{c} P_{i\times j}=f_{i\times j}\cdot \lambda_{i}. \end{array}$$

So *k* groups of *P* values can be obtained. However, since the number and type of position information of basis space components obtained between different groups are uncertain, the sum of *P* values between different groups with the same position of basis space components is required. The size of the final sum represents the amount of information contained by each lipid in the original data. The sum operation is shown in Equation (15).

(15) $$\begin{array}{c} Q_{j}=\overset{k}{\underset{i=1}{\sum }}p_{i\times j}. \end{array}$$

Using the above method, the types of lipids that have a greater impact on acne in the original data can be determined.

## 3. Results

### 3.1. The Experiment Results and Analysis of PCA and KPCA Methods

The PCA or KPCA method only can test DS, HS, and NC samples, respectively. We can determine the number of principal components based on the cumulative contribution rate. The lipids which have great influence on the samples can be found using the corresponding eigenvalues and eigenvectors. In Figure 2 the Venn diagram is used to show the similarities and differences on the experimental results of DS, HS, and NC samples, i.e., the lipids which have larger influence on the samples, using the PCA and KPCA methods when the cumulative contribution rate is 95%. The numbers in Figure 2 represent the labels of some certain lipids, and the descriptions of the lipids are presented in Table 1.

In Figure 2(a), it is found that three lipids such as numbers 1311, 1264, and 1240 have the greater impact on the DS samples not only using PCA but also KPCA methods. In Figure 2(b), the lipid like number 608 which has the larger influence on the HS samples is found using PCA and KPCA methods. Besides, another lipid number 607 is also found using the PCA method, and 2 lipids like number 2334 and number 776 are found using the KPCA method. In Figure 2(c), the same 7 lipids have a significant effect on NC samples by not only PCA but also KPCA. In Figure 2, the contribution of the lipid decreases along the direction of arrow step by step.

Figure 3 shows the lipids which have the larger influence on the samples when the cumulative contribution rate is 99%, and Figures 3(a)–3(c) are the results of PCA and KPCA on DS, HS, and NC samples, respectively. The lipids' specific description is shown in Table 2.

It can be seen from Figure 3 that 9 lipids including numbers 1311, 1264, 1240, 1205, 1245, 1266, 1236, 1315, and 1283 have the larger influence on DS samples by both PCA and KPCA. For HS samples, the similar results are obtained. Five lipids like numbers 608, 2334, 776, 2172, and 607 which contribute to the status of samples are obtained using KPCA, and among these, 4 lipids are results of PCA. For NC samples, the same results obtained by PCA and KPCA are gotten including 14 lipids. And some differences can be seen from Figure 3(c). For example, number 2374 is found by PCA, and number 889 is found by KPCA.

Furthermore, both PCA and KPCA can be used to find the primary lipids which contribute to the status of different samples. KPCA, however, can obtain more complete and richer lipids than PCA, because it can mine nonlinear information in the original data. In addition, the lipids which have the main influence on the HS samples such as numbers 608, 2334, and 776 are completely different from DS and NC samples and can be used as an indicator of the improvement of skin status during the course of acne treatment. For the DS and NC samples, some lipids are found simultaneously like numbers 1311, 1264, and 1240. It is shown that these lipids are significant both for DS samples and NC samples. At the same time, some differences appear. For example, some lipids like numbers 1304, 1279, and 1302 only exist in the results of NC samples. It suggests that when these lipids are rich, the status of skin is very healthy and could effectively suppress the growth of toxin.

### 3.2. The Experimental Results and Analysis of MCCA Method

PCA and KPCA methods can only analyze one kind of sample set. In order to simultaneously analyze three kinds of sample sets and to obtain lipids which can distinguish DS, HS, and NC samples, MCCA is used. Experiments show that 19 lipids as shown in Table 2 which bear on all sample sets DS, HS, and NC are obtained. Among the 19 kinds of lipids, 13 lipids exert different effects on the three types of sample sets. As shown in Figure 4, the abscissa represents the samples, and the ordinate denotes the influence degree, i.e., the contents of the lipids. The descriptions of the found lipids are presented in Table 3.

It can be concluded from Figure 4 that the lipids with different effects on these three samples sets can be categorized into three types, respectively, shown in Figures 4(a)–4(c). Among of three line charts, Figure 4(a) reveals that all samples follow the same variation trend under the influence of the lipids like No. 1219, No. 1264, and No. 1311. For DS and HS samples, difference of lipids contents is puny. For NC, however, obvious decrease appears. Therefore, No. 1219, No. 1264, and No.1311 can be used to distinguish DS and HS sample sets from NC sample set.

Figure 4(b) demonstrates six lipids (No. 1061, No. 1200, No. 1240, No. 1266, No. 1302, and No. 1315) with the effects on the three sample sets. These six representative lipids have greater impact on DS samples compared with HS and NC and have little effects difference on the latter two. It can be inferred that when the contents of these six lipids are small, the status of skin on DS samples is improving or that skin is involved in a sound condition.  Figure 4(c) depicts the impact of four kinds of lipids (No. 1205, No. 1236, No. 1245, and No. 1304) on the samples which are a monotonic decrease trend for DS, HS, and NC samples. Thus, these four lipids can be taken as metrics to distinguish DS, HS, and NC.

The content of lipids of samples fluctuates only in response to certain lipids as shown in Figures 5–7. For example, No. 95, No. 1069, and No. 1108 influence DS samples alone, No. 608, No. 2172, and No. 2334 only effect on HS samples, and No. 889 and No. 2374 only affect NC samples.

Figure 5 shows different content of lipids like No. 95, No. 1069, and No. 1108 for DS, HS, and NC samples. The abscissa is the sample number, and the ordinate is the content of the lipids. As demonstrated above, these three lipids only have a major impact on DS, and thus, the content in DS is obviously higher than that in the other two samples. We can safely conclude that when the content of these three lipids increases significantly, the skin of the subject is in a diseased condition and needs treatment. Conversely, if a patient with acne undergoes a dramatic decrease on the content of these lipids during treatment, it demonstrates that the skin condition is turning better.

Likewise, Figure 6 shows the content changes of lipids like No. 608, No. 2172, and No. 2334 for DS, HS, and NC. These three lipids are absent for DS and NC while they are a marked increase for HS. The result suggests that when the content of lipids like No. 608, No. 2172, and No. 2334 escalates, the subjects' skin is during a transitional period.

Figure 7 presents two lipids such as No. 889 and No. 2374 which have effects only on NC sample sets. It can be seen that the content of these two lipids in NC increases notably while is rather low in DS and HS. If the content of No. 889 and No. 2374 rises significantly in the process of treatment, it indicates that the treatment is effective and the skin is in a healthy condition.

## 4. Conclusion

As one of the common skin diseases in the world, acne has a large number of patients with complex etiology and will cause certain psychological and physiological damage to patients. Therefore, the research and treatment of acne is of great significance. In this paper, the pathogenesis of acne is analyzed from the perspective of metagenomics. In view of the large amount of data on acne metagenomics, it is found that it is difficult to find the hidden valuable data. And the method of machine learning is proposed for analysis. In the experiment, PCA, KPCA, and MCCA are used to analyze the data of DS, HS, and NC sample sets, and the lipids that can distinguish the three sample sets are obtained. Comparing all experimental results, it is found that the lipid of No. 1240 can be used to distinguish DS sample set, lipids like No. 608 and No. 2334 can be used to distinguish HS sample set, and lipids that can be used to distinguish NC sample set are No. 1264 and No. 1311. It can be concluded from the experimental results that the method of machine learning can quickly and accurately determine and distinguish lipids in different sample sets, which can provide certain auxiliary guiding significance for the prevention, diagnosis, and treatment of acne.

## Figures and Tables

**Figure 1:** The framework of the proposed method.

**Figure 2:** The lipids with larger contributes to (a) DS samples, (b) HS samples, and (c) NC samples when the cumulative contribution rate is 95%.

**Figure 3:** The lipids with larger contributes to (a) DS samples, (b) HS samples, and (c) NC samples when the cumulative contribution rate is 99%.

**Figure 4:** Lipids with different effects on DS, HS, and NC sample sets.

**Figure 5:** Lipids with effects only on DS sample set: (a) No. 95, (b) No. 1069, and (c) No. 1108.

**Figure 6:** Lipids with effects only on HS sample set: (a) No. 608, (b) No. 2172, and (c) No. 2334.

**Figure 7:** Lipids with effects only on NC sample set: (a) No. 889 and (b) No. 2374.

**Table 1:** The specific descriptions of the lipids shown in Figure 1.

Label	Description
607	PC (20 : 0/21 : 0)
608	PC (20 : 0/26 : 0)
776	PC (34 : 0/16 : 0)
1205	1-(6-[5]-Ladderane-hexanoyl)-2-(8-[3]-ladderane-octanyl)-sn-glycerophosphocholine
1236	1-(8-[3]-Ladderane-octanoyl)-2-(8-[3]-ladderane-octanyl)-sn-glycerophosphoethanolamine
1240	PS (22 : 6 (4Z, 7Z, 10Z, 13Z, 16Z, 19Z)/18 : 1(9Z))
1245	1-(8-[3]-Ladderane-octanoyl)-2-(8-[3]-ladderane-octanyl)-sn-glycerophosphoethanolamine
1264	PS (22 : 6 (4Z, 7Z, 10Z, 13Z, 16Z, 19Z)/19 : 1(9Z))
1266	1-(6-[3]-Ladderane-hexanoyl)-2-(8-[3]-ladderane-octanyl)-sn-glycerophosphocholine
1311	PS (22 : 6 (4Z, 7Z, 10Z, 13Z, 16Z, 19Z)/19 : 0)
2334	GlcAbeta-Cer (d18 : 1/18 : 0)

**Table 2:** Lipids with effects on all sample sets (DS, HS, and NC), obtained by MCCA.

Label	Description
1061	Tacrolimus
1192	FMC-5 (d18 : 1/18 : 0)
1200	PS (22 : 6 (4Z, 7Z, 10Z, 13Z, 16Z, 19Z)/19 : 0)
1205	1-(6-[5]-Ladderane-hexanoyl)-2-(8-[3]-ladderane-octanyl)-sn-glycerophosphocholine
1219	PG (20 : 3(8Z, 11Z, 14Z)/17 : 0)
1236	1-(8-[3]-Ladderane-octanoyl)-2-(8-[3]-ladderane-octanyl)-sn-glycerophosphoethanolamine
1240	PS (22 : 6 (4Z, 7Z, 10Z, 13Z, 16Z, 19Z)/18:1(9Z))
1244	PS (20 : 5(5Z, 8Z, 11Z, 14Z, 17Z)/20 : 0)

**Table 3:** Lipids with effects on single sample set, obtained by MCCA.

Label	Description
95	Prodelphinidin B6
608	PC (20 : 0/26 : 0)
889	PS (20 : 2(11Z, 14Z)/21 : 0)
1069	PS (18 : 4(6Z, 9Z, 12Z, 15Z)/22 : 2(13Z, 16Z))
1108	PS (20 : 3(8Z, 11Z, 14Z)/19 : 0)
2172	1-(10-Methylhexadecanyl)-2-(8-[3]-ladderane-octanyl)-sn-glycerophosphocholine
2334	GlcAbeta-Cer (d18:1/18 : 0)
2374	Phoenicoxanthin/adonirubin/3-hydroxycanthaxanthin

## Data Availability

Data are not convenient to be published because the related agreement has been signed with the partner in this study.
